The article "A Comparison of Dynamic and Static Hip-Knee-Ankle Angle during Gait in Knee Osteoarthritis Patients and Healthy Individuals" was published in 2021. Journal: Appl Bionics Biomech.

# A Comparison of Dynamic and Static Hip-Knee-Ankle Angle during Gait in Knee Osteoarthritis Patients and Healthy Individuals

**DOI:** 10.1155/2021/6231406

**Published:** 2021-11-22

**Authors:** Li Zhang, Geng Liu, Bing Han, Yuzhou Yan, Junhua Fei, Jianbing Ma, Yunfei Zhang

**Affiliations:** ^1^Innovation Center of Bioengineering, Shaanxi Engineering Laboratory for Transmissions and Controls, Northwestern Polytechnical University, Xi'an 710072, China; ^2^Honghui Hospital, Xi'an Jiaotong University College of Medicine, Xi'an 710054, China; ^3^Tangdu Hospital, Air Force Medical University, Xi'an 710038, China

## Abstract

Malalignment of the lower limbs is the main biomechanical factor for knee osteoarthritis (KOA). The static hip-knee-ankle angle (S-HKAA) measured from radiograph is regarded as the “gold standard” of the malalignment. However, many evidences showed that the S-HKAA has no significant correlation with the knee dynamic-load distribution, unlike the dynamic HKAA (D-HKAA). The purpose of this study was to quantitatively analyze the D-HKAA and investigate the relationship between D-HKAA and S-HKAA for both KOA and healthy participants. In this paper, twenty-five healthy subjects and twenty-five medial compartment KOA (M-KOA) patients were recruited. Three-dimensional motion analysis and standing lower-limbs-full-length radiograph were utilized to obtain the D-HKAA and S-HKAA, respectively. The results showed that the mean D-HKAA was more varus than the S-HKAA (*p* < 0.05). For the mean D-HKAA, larger varus angle was observed in swing phase than stance phase (*p* < 0.05). Compared with healthy subjects, the M-KOA patients had remarkably smaller S-HKAA and D-HKAA during gait cycle (*p* < 0.01). For the relationship between the S-HKAA and mean D-HKAA, no significant correlation was found for both healthy subjects and M-KOA patients (*r* < 0.357, *n* = 25, *p* > 0.05, Spearman correlation analysis). In conclusion, the S-HKAA was limited to predict the D-HKAA for both M-KOA patients and healthy subjects. The D-HKAA should be given more attention to the orthopedist and the designer of knee brace and orthotics.

## 1. Introduction

Knee osteoarthritis (KOA), as the fourth leading disabling disease, is a significant public health problem [1–3]. Epidemiological studies show that approximately 7-17% of individuals will present with KOA [4–7]. Malalignment of the lower limbs is the main factor for the initiation and progression of KOA, which changes the knee adduction moment and then results in the abnormal load distribution between knee medial and lateral compartment [7–9].

As the “gold standard” measure of the malalignment, hip-knee-ankle angle (HKAA) measured from a standing lower-limbs-full-length anterior-posterior radiograph provides important guidance for the preoperative diagnosis of orthopedists, surgical planning and assessment of total knee arthroplasty (TKA), design of brace and orthotics, and so on [10–12]. However, some studies pointed out that there was no significant correlation between static HKAA (S-HKAA) and dynamic load distribution of knee joint, which mainly because the S-HKAA was limited to predict the dynamic behavior [13–16]. As an advanced and cutting-edge method, dynamic HKAA (D-HKAA) obtained from gait analysis can accurately and real-time reflect the loading condition of the knee joint and is increasingly used in clinical work [15–18].

In the past few years, in order to study the D-HKAA and analyze the relationship between D-HKAA and S-HKAA, a few related researches have been done. Larose et al. [13] investigated the correlation between static radiographic alignment and dynamic motion-capturing alignment during gait for TKA postoperative patients. They pointed out that there was a weak relationship between static and dynamic alignment. Clement et al. [18] studied whether the S-HKAA was predictive of D-HKAA throughout the gait cycle for healthy people. The results showed that the relationship between S-HKAA and D-HKAA was moderate for varus knee and negligible for valgus knee. Riviere et al. [15] compared the static alignment with dynamic alignment during stance phase on patients after TKA. They found that the S-HKAA had a moderate relationship with the mean D-HKAA of stance phase.

However, all of the researches mentioned above were only for post-TKA patients or healthy subjects. To our knowledge, no previous study has quantitatively analyzed the D-HKAA and studied the relationship between D-HKAA and radiograph-based S-HKAA for both medial compartment KOA (M-KOA) patients and healthy subjects during gait. Although Duffell et al. [19] analyzed the differences between S-HKAA and D-HKAA in healthy subjects and KOA patients, the proposed S-HKAA was obtained by using a motion capture system rather than standing lower-limbs-full-length radiograph which was commonly used in medical field.

Therefore, the purpose of this study was twofold. The first purpose was to quantitatively analyze the D-HKAA during gait for both KOA patients and healthy subjects. And the differences of mean D-HKAA and S-HKAA, the mean D-HKAA in different gait phases, and the mean D-HKAA of KOA patients and healthy subjects were explored. The second purpose was to investigate the corrections between D-HKAA and S-HKAA during different phases for both KOA patients and healthy subjects. It was hypothesized that the mean D-HKAA would be smaller (more varus) than the S-HKAA and the mean D-HKAA of swing phase would be smaller (more varus) than that of stance phase for both KOA patients and healthy subjects. The S-HKAA was no significant correlated with the mean D-HKAA for both the healthy subjects and M-KOA patients.

## 2. Methods

### 2.1. Subjects

Twenty-five patients (11 males and 14 females, age: 55 ± 12 yrs., height: 165.1 ± 7.8 cm, mass: 71.4 ± 3.9 kg, and BMI: 25.9 ± 5.8 kg/m^2^) clinically diagnosed with M-KOA by orthopedists and twenty-five healthy subjects (15 males and 10 females, age: 23 ± 8 yrs., height: 174.8 ± 5.2 cm, mass: 69.9 ± 5.8 kg, and BMI: 23.1 ± 4.7 kg/m^2^) were recruited in this study. In total, 100 lower limbs (bilateral lower limbs) were analyzed in this study. Exclusion criteria were any previous history of lower-limb injuries, any other neuromuscular disease and a BMI > 35 kg/m^2^ for all participants, and the inability to fulfill the experiment, rheumatoid arthritis, and unilateral or bilateral lateral compartment KOA for M-KOA patients. This study had ethical approval from the Human Research Ethics Committee of our university. All recruited participants provided written informed consent prior to the experiments.

### 2.2. Radiographic Data Acquisition and Processing

A standing lower-limbs-full-length anterior-posterior radiograph was captured by one radiographer for all participants. To ensure that the patella was in the center of the femoral condyles, the participant was asked to stand with a forward knee position [20]. As shown in Figure 1, the S-HKAA was obtained by drawing lines connecting the hip, knee, and ankle joint centers. The hip, knee, and ankle joint centers were defined as the center of the femoral head, the midpoint of the femoral epicondyles, and the midpoint of the medial and lateral malleolus, respectively. All S-HKAA data were measured by one orthopedist. Reliability of the S-HKAA measurement (intraclass correlation coefficient (ICC) = 0.995; 95%confidence interval (CI) = 0.994, 1) has already been reported [21].

### 2.3. Gait Data Acquisition

The gait data acquisition was conducted on the same day as the radiographic data acquisition. As shown in Figure 2(a), a ten-camera motion capture system (Vicon version 3.3, Vicon Motion Analysis Inc., Oxford, UK) was utilized to capture 3-dimensional (3D) kinematic data of participant's lower limbs. Fifty-five hemispherical reflective markers (15 mm) were attached to the full-body of the participant according to the Vicon-gait marker set model. The sampling frequency of the motion capture system was set to 100 Hz. A three-force-platforms system (BP 600600, AMTI, Watertown, MA, USA) embedded in the laboratory floor was used to capture 3D ground reaction forces (GRFs). The sampling frequency of the force platforms system was set to 1000 Hz. During the experimental session, the participant was asked to walk at a self-selected speed on a 15 m walkway after an upright standing calibration process. The middle 10 gait cycles of the 15 m walkway were used for data analysis. For each participant, 20 repeated trials (more than 200 repeated gait cycles) were performed. To remove the effects of fatigue, a 1 min rest period was provided between two sessions.

### 2.4. Gait Data Processing

All of the simulation processes were performed in OpenSim software (OpenSim version 3.3, SimTK, Stanford, CA, USA). A musculoskeletal model (3DGaitModel 2392) possessed 23 degree-of-freedom (DOF) and 92 muscles (mainly lower limb muscles) was employed to analyze the gait data (as shown in Figure 2(b)). Before all of the process, a 4th-order Butterworth filter with 6 Hz cut-off frequency was used for the data of marker coordinates and GRFs.

The simulation process could be summarized as scale, IK (inverse kinematics), ID (inverse-dynamics), RRA (residual reduction algorithm), and PKA (point kinematics analysis). Firstly, scale was performed by changing model's anthropometry so that it matched the participant as closely as possible, based on the differences between marker data of upright standing calibration and the musculoskeletal model. Then, IK and ID were utilized to fulfill kinematic and dynamics simulation of human body, respectively. To further reduce the motion errors between model and participant, RRA was adopted by adjusting the kinematics and torso mass center of participant's model and getting dynamically consistency between the kinematics and GRFs. Finally, the 3D kinematic data of hip, knee, and ankle joint centers were computed by used PKA (as shown in Figure 2(c)). The definitions of the joint centers were the same as those defined on the radiographic data. The D-HKAA was obtained by projecting the 3D kinematic data into the coronal plane and computing using Python software (Python version 3.7). Reliability of the similar D-HKAA measurement (intraclass correlation coefficient (ICC) = 0.82; 95%confidence interval (CI) = 0.59, 0.92) has already been reported [22].

Mean D-HKAA curves were computed by averaging the 200 repeated gait cycles in each subject. The D-HKAA curves were normalized from 0% to 100% of the average gait cycle (from heel strike to next heel strike of the same foot).  Figure 3 shows the typical S-HKAA and D-HKAA curves of one healthy subject and one M-KOA patient. For comparing the differences among different gait phases, the curves could be divided into two phases: stance phase and swing phase. And the curves of the stance phase could be further divided into three subphases: initial, middle, and terminal stance subphase [3, 23]. For analyzing the differences quantitatively, the mean value of D-HKAA and the mean differences between S-HKAA and D-HKAA for each phase were computed.

### 2.5. Statistical Analysis

A standardized coefficient of variation (SCV) was used to assess the reproducibility of measured parameters. The SCV is determined by normalizing the coefficient of variation (CV) with the range of variations of the parameters in the present sample population [24–26], that is defined as follows:

(1) $$\begin{array}{c} \text{SCV}=\frac{\text{CV}∙\text{MEAN}}{4∙\text{SD}}, \end{array}$$

where MEAN and SD are the mean and standard deviation (SD) of the measured parameter. CV is defined as:

(2) $$\begin{array}{c} \text{CV}=\sqrt{\frac{\sum_{i=1}^{n}{{\text{CV}}_{j}}^{2}}{n}}∙100\%, \end{array}$$

where CV_*j*_ is the ratio of the SD of the measurement performed on sample *j* to mean of this measurement.

All data were expressed as mean ± SD. The distributions were checked for normality using Kolmogorov-Smirnov test before statistical analyses [27]. Due to relatively small number of samples, the nonparametric Wilcoxon signed-rank test was used for the statistical comparisons [28, 29]. The Spearman correlation analysis was chosen to study the association between S-HKAA and mean D-HKAA for both healthy subjects and M-KOA patients. According to the effect sizes reported by Clement et al. [18], to achieve power of 0.8 with *α* at 0.05, the sample size required for HKAA is fifteen. Statistical analyses were performed using the Statistical Package for Social Sciences (SPSS version 16, SPSS Inc., Chicago, IL, USA) software.

## 3. Results

Figure 4 shows the S-HKAA and mean D-HKAA for both healthy subjects and M-KOA patients. In general, the M-KOA patients had significantly lower (more varus) mean D-HKAA during the whole gait cycle (167.2 ± 3.3° vs. 174.1 ± 2.8°), stance phase (169.1 ± 2.2° vs. 175.8 ± 2.1°), and swing phase (165.9 ± 3.7° vs. 169.2 ± 3.2°) than the healthy subjects, which was accord with the result of S-HKAA (171.2 ± 2.3° vs. 178.3 ± 1.7°) (*p* < 0.01).

As shown in Figures 4(a) and 4(b), the mean D-HKAA of the whole gait cycle, stance phase, and swing phase was significantly lower (more varus) than the S-HKAA for both healthy subjects and M-KOA patients (*p* < 0.01). Compared to the S-HKAA (healthy subjects: 178.3 ± 1.7°, M-KOA patients: 171.2 ± 2.3°), the mean D-HKAA of the whole gait cycle, stance phase, and swing phase was 4.2 ± 2.6° (174.1 ± 2.8°), 2.5 ± 1.9° (175.8 ± 2.1°), and 9.1 ± 2.8° (169.2 ± 3.2°) lower (more varus) for healthy subjects, and 4.0 ± 2.9° (167.2 ± 3.3°), 2.1 ± 2.3° (169.1 ± 2.2°), and 5.3 ± 3.4° (165.9 ± 3.7°) lower (more varus) for M-KOA patients, respectively. For the mean D-HKAA, the swing phase had significantly lower (more varus) mean value and larger standard deviation than the stance phase (*p* < 0.05) (as shown in Figure 4(b)). Compared to the stance phase, the standard deviation of D-HKAA and the differences between mean D-HKAA and S-HKAA during swing phase increased by 47.4% and 264.1% for healthy subjects and 47.8% and 152.4% for M-KOA patients, respectively. As shown in Figure 4(c), for all participants, the mean D-HKAA of terminal stance subphases was significantly lower (more varus) than that of initial and middle stance subphase (*p* < 0.05). But there was no significant difference between mean D-HKAA of initial and middle stance subphase (*p* > 0.05). Compared to the S-HKAA, the D-HKAA of initial, middle, and terminal stance subphase was 3.1 ± 1.7° (175.2 ± 1.6°), 2.2 ± 1.9° (176.1 ± 1.9°), and 4.5 ± 2.3° (173.8 ± 2.4°) lower (more varus) for healthy subjects and 2.6 ± 2.0° (168.6 ± 1.8°), 1.3 ± 2.2° (169.9 ± 2.1°), and 3.4 ± 2.6° (167.8 ± 2.7°) lower (more varus) for M-KOA patients. Compared to the initial and middle-stance phase, the deviation between mean D-HKAA and S-HKAA during the terminal stance subphase increased by 45.2% and 104.5% for healthy subjects and 30.8% and 161.5% for M-KOA patients, respectively.

For healthy subjects, the SCVs were 1.1%, 5.3%, 3.8%, and 7.4% for S-HKAA, D-HKAA of whole gait cycle, D-HKAA of stance phase, and D-HKAA of swing phase, respectively. For KOA patients, the SCVs were 1.3%, 6.2%, 4.4%, and 7.9% for S-HKAA, D-HKAA of whole gait cycle, D-HKAA of stance phase, and D-HKAA of swing phase, respectively.

Table 1 shows the results of Spearman correlation analysis between S-HKAA and mean D-HKAA for both healthy subjects and M-KOA patients. For the healthy subjects, the S-HKAA in the healthy subjects presented a no significant correlation (*n* = 25, *p* > 0.05) with the mean D-HKAA of whole gait cycle (*r* = 0.326), stance phase (*r* = 0.291), and swing phase (*r* = 0.357). During the stance phase of healthy subjects, there were no significant correlations (*n* = 25, *p* > 0.05) between S-HKAA and mean D-HKAA of initial (*r* = 0.282), middle (*r* = 0.294), and terminal (*r* = 0.335) stance subphase. For the M-KOA patients, the S-HKAA was no significant correlated (*n* = 25, *p* > 0.05) with the mean D-HKAA of whole gait cycle (*r* = 0.247), stance phase (*r* = 0.216), and swing phase (*r* = 0.261). During the stance phase of M-KOA patients, there were no significant correlations (*n* = 25, *p* > 0.05) between S-HKAA and mean D-HKAA of initial (*r* = 0.198), middle (*r* = 0.220), and terminal (*r* = 0.258) stance subphase. In total, the S-HKAA was limited to predict the D-HKAA for both M-KOA patients and healthy subjects.

## 4. Discussion

The S-HKAA measured from a standing lower-limbs-full-length anterior-posterior radiograph is regarded as the “gold standard” measure of the malalignment for the preoperative diagnosis of orthopedists, surgical planning and assessment of TKA, design of brace and orthotics, and so on. However, some researchers highlighted that the S-HKAA was insufficient to predict the dynamic loading behavior of knee joint and then study or treatment KOA, unlike the D-HKAA. Therefore, this research is aimed at studying the D-HKAA during gait, analyzing the relationship between D-HKAA and S-HKAA, and comparing the D-HKAA and the relationship between M-KOA patients and healthy subjects.

We found that there was a significant difference between D-HKAA and S-HKAA (the D-HKAA was smaller (more varus) than the S-HKAA) for both the healthy subjects (4.2 ± 2.6°) and M-KOA patients (4.0 ± 2.9°) (*p* < 0.01). These differences could explain from two reasons mainly. First, the real knee joint has internal-external rotation in the horizontal plane. During the knee flexion-extension motion, the tibia rotates around the femoral condyles [30]. In the sagittal plane, the real knee joint moves with a polycentric motion during gait, whereby the center of rotation changes during the rotation [31, 32]. Since the nonuniform shape of the knee articular surface and the complicated physical structure of the femur and tibia, the femur and tibia can be approximated as a bielliptical structure [30]. During the knee flexion-extension motion, the tibia rolls on femur resulting in anterior-posterior (A-P) translation [33]. Overall, during the gait motions, the relative rotation between tibia and femur resulted in the change of the flexion-extension axis, which directly affected the value of D-HKAA. Second, there are many soft tissues envelope the knee joint, which can restrict the range of motion (ROM) and maintain joint stability. For example, the tibial-fibular collateral ligaments (TCL/FCL) mainly restrain the varus-valgus stress placed on the knee joint and limit the internal-external rotation [34, 35]. The anterior-posterior cruciate ligaments (ACL/PCL), located within the joint capsule and crossed each other obliquely, mainly prevent the anterior-posterior translation and limit the hyperextension and internal-external rotation [36, 37]. And patellar ligament (PL) primarily assists the knee extension [38, 39]. However, the soft tissues not completely restrict the motion of knee joint in frontal plane, and the laxities of knee joint are more or less exist, which are potentially partly resulted in the change of D-HKAA. The value of S-HKAA showed that there was an inherent knee varus for all the participants (healthy subjects: 178.3 ± 1.7°, M-KOA patients: 171.2 ± 2.3°). During the gait cycle, the changing loading condition could lead to an increase of knee varus, which might decrease the D-HKAA.

Our results showed that the D-HKAA of swing phase had significantly lower (more varus) mean value and larger standard deviation than the stance phase for both the healthy subjects (169.1 ± 2.2° vs. 165.9 ± 3.7°) and M-KOA patients (175.8 ± 2.1° vs. 169.2 ± 3.2°) (*p* < 0.05). As shown in Figure 5, compared with the stance phase, the ROM of swing phase was increased about 2 times for KOA patients and 1.5 times for healthy subjects. Previous studies have reported that there was a small A-P translation when the flexion-extension angle of knee joint was less than 20 deg, but an increased A-P translation (>19 mm) when the rotation angle of knee joint increased [37–40]. During the swing phase, the larger A-P translation and internal-external rotation could result in a smaller mean value and larger standard deviation of D-HKAA. The results of our study indicated that the mean D-HKAA of terminal stance subphase was significantly lower (more varus) than that of initial and middle stance subphase for both the healthy subjects (175.2 ± 1.6, 176.1 ± 1.9° vs. 173.8 ± 2.4°) and M-KOA patients (168.6 ± 1.8°, 169.9 ± 2.1° vs. 167.8 ± 2.7°) (*p* < 0.05). But there was no significant difference between mean D-HKAA of initial and middle stance subphase (*p* > 0.05). This result also could be explained by the larger knee ROM during terminal stance subphase compared with initial and middle stance subphase. Our results also pointed out that the M-KOA patients had significantly lower (more varus) S-HKAA (171.2 ± 2.3° vs. 178.3 ± 1.7°) and mean D-HKAA (167.2 ± 3.3° vs. 174.1 ± 2.8°) than the healthy subjects (*p* < 0.01). As shown in Figure 5, the results could be explained by a large difference of knee ROM between M-KOA patients and healthy subjects (55.1 ± 2.1° vs. 64.9 ± 2.8°).

Clinically, a radiation-free method to measure dynamic alignment would be very useful, as this would be a good indicator for kinematically alignment TKA which is aimed at restoring the dynamic motion and function of knee joint. The clinical disadvantage of static standing alignment was their poor relationship with the survivorship of TKA [15]. This poor relationship could be explained by poor correlation between static standing alignment and dynamic motion and function of knee joint. In this paper, we found that there were no significant correlations between S-HKAA and mean D-HKAA for both healthy subjects (*r* = 0.326, *n* = 25, *p* > 0.05) and M-KOA patients (*r* = 0.247, *n* = 25, *p* > 0.05) (Spearman correlation analysis). These results agreed with the finding of Rivieve et al. [15], Clement et al. [18], and Inan et al. [41]. Rivieve et al. [15] showed no significant correlation between the S-HKAA and D-HKAA (*r* = 0.14, *n* = 35, *p* = 0.449, Pearson correlation analysis), but it was only on patients after TKA. Clement et al. [18] found the S-HKAA had a low coefficient with D-HKAA (*r* = 0.266, *n* = 90, *p* = 0.001, Pearson correlation analysis) for healthy subjects. Inan et al. [41] pointed out that the relationship between standing alignment and dynamic lower extremity alignment was poor for children with achondroplasia (*p* > 0.05, *n* = 13, Spearman correlation analysis), but unfortunately, they did not report the value of *r*. Therefore, it seemed that the S-HKAA was insufficient to predict the D-HKAA and then dynamic motion and function of knee joint for both healthy subjects and M-KOA patients. These observations could explain why several researchers found that there was a poor relationship between static standing alignment and survivorship of TKA.

A number of limitations associated with this study are worth discussing. Firstly, the soft tissue artifacts possibly existed in the gait experiment. In this study, multiple methods were utilized to reduce the soft tissue artifacts, such as placing the markers on the bony landmarks as much as possible and twenty repeated tests for each participant. Secondly, the number of the M-KOA patients recruited in this study was relatively small. More M-KOA patients will be recruited in the future. Finally, only gait experiment was carried out in this study. Because the different motions possessed different kinematics, the results of this study were only suitable for gait and not for other motions. Quantitative analyzing the D-HKAA and investigating the relationship between D-HKAA and S-HKAA during other motions, such as running, stair climbing and sit-stand-sit, will be studied in the future.

## 5. Conclusions

In this study, the D-HKAA and S-HKAA of M-KOA patients and healthy subjects during gait were analyzed and compared. Based on the experimental results, the main conclusions can be summarized as follows:

1. The D-HKAA was significant more varus than the S-HKAA, and the mean D-HKAA of swing phase was significantly more varus than that of stance phase due to the larger ROM of knee joint during gait cycle, especially in swing phase
2. Because of the differences of knee ROM between M-KOA patients and healthy subjects, the S-HKAA and D-HKAA was smaller for M-KOA patients than healthy subjects during gait cycle
3. The S-HKAA was no significantly correlated with the mean D-HKAA for both the healthy subjects and M-KOA patients. The changes of cartilage morphology and soft tissue mechanical properties after KOA could reduce the correlation between S-HKAA and D-HKAA

Overall, for both M-KOA patients and healthy subjects, the S-HKAA measured from a standing lower-limbs-full-length radiograph was limited to predict the D-HKAA. The D-HKAA obtained from gait analysis should be given more attention to the orthopedist and the knee brace and orthotics designer.

## Figures and Tables

**Figure 1:** Standing lower-limbs-full-length anterior-posterior radiographs of healthy subjects (a) and medial compartment knee osteoarthritis (M-KOA) patients (b). Static hip-knee-ankle angle (S-HKAA) was obtained by drawing lines connecting the hip, knee, and ankle joint centers. The hip, knee, and ankle joint centers were defined as the center of the femoral head, the midpoint of the femoral epicondyles, and the midpoint of the medial and lateral malleolus, respectively.

**Figure 2:** Gait experiment and dynamic data processing: (a) gait experiment, (b) musculoskeletal simulation model, and (c) dynamic hip-knee-ankle angle (D-HKAA).

**Figure 3:** Typical S-HKAA (dash line) and D-HKAA (mean: solid line and SD: shading) curves during gait cycle of healthy subject (red line) and M-KOA patient (blue line) (The vertical red and blue shading represent the boundaries between stance and swing phase, initial and middle stance subphase, and middle and terminal stance subphase for healthy subjects and M-KOA patients, respectively.)

**Figure 4:** S-HKAA and mean D-HKAA for healthy subjects and M-KOA patients, A S-HKAA and mean D-HKAA of whole gait cycle, B D-HKAA of stance phase and swing phase, and C D-HKAA of initial, middle, and terminal stance subphase.

**Figure 5:** Knee joint angle curves of healthy subjects (mean: red solid line and SD: red shading) and M-KOA patients (mean: blue dash line and SD: blue shading) during gait (The vertical red and blue shading represent the boundary between stance phase and swing phase for healthy subjects and M-KOA patients, respectively.)

**Table 1:** The results of correlation analysis between S-HKAA and mean D-HKAA for both the healthy subjects and M-KOA patients.

Subjects	*r*/*p*	Whole gait cycle	Stance phase	Swing phase	Initial stance subphase	Middle stance subphase	Terminal stance subphase
Healthy subjects (*n* = 25)	*r*	0.326	0.291	0.357	0.282	0.294	0.335
	*p*	0.132	0.115	0.144	0.113	0.126	0.137
M-KOA patients (*n* = 25)	*r*	0.247	0.216	0.261	0.198	0.220	0.258
	*p*	0.206	0.184	0.234	0.179	0.188	0.215

## Data Availability

The data used to support the findings of this study are available from the corresponding author upon request.
